# A Quantitative Analysis of Country Relations in Foreign Direct Investment

**DOI:** 10.1155/2022/4144073

**Published:** 2022-04-15

**Authors:** Huawei Fu, Li Yan, Hua Li

**Affiliations:** ^1^School of Economics and Management, Xidian University, Xi'an 471000, China; ^2^Department of Administrative Sciences, University of Quebec, Ottawa, Canada

## Abstract

According to Dunning's eclectic theory, the location advantages play a key role in international investment mode choice, in which the country relations are important determinants. In some previous studies, the country relations and another bilateral factor, the country distance, are often confused, which can result in the inconsistency of conclusions. And excepting political factors, the economic dependence and other relations are insufficiently considered in the literature. This article makes a distinction between relation and distance, and puts forward a simplified analytical framework, the indicator system, and some quantitative methods for country relations. The indicators, including political, economic, and social factors, can better satisfy the horizontal analysis of the outbound investment. The economic and social indicators are determined by the magnitude of interaction as well as the share in the home country, and hence, the evaluation results can reflect the differences between the two countries. Finally, by evaluating the relations of other BRICS countries with China, the rationality is illustrated.

## 1. Introduction

In the literature of location choice of outbound investment, many authors analyzed factors such as the foreign capital policy, economic development level, market size, infrastructure, resource endowment, trade barriers, labor force, and cost in foreign markets based on the eclectic theory of international market proposed by Dunning [1–4]. In reality, it is a fact often observed that outbound investment and other forms of economic cooperation do not uniquely depend on the unilateral environment of the host country. Indeed, the investment behavior may be found paradoxical sometimes if only the investment environment in the host country is taken into account. Buckley et al. [5] found in their empirical analysis that China's investment would flow into the high political risk areas. Kolstad and Wiig [6] found that China's foreign direct investment outflows tend to seek rich natural resources in weak constitutional system countries. And Ramasamy et al. [7] also found that China's state-owned enterprises do not avoid high political risk in a perspective of enterprise. This seems an irrational risk attitude. The authors ascribe this to the strategic motivation of the Chinese government and believe that existing theories need to be developed to explain such phenomena. The search for resources of Chinese outward foreign direct investment (OFDI) is understandable because China has been the largest manufacturing country for a long time. However, it is impossible for China to ignore high political risks in its strategic considerations. In fact, strategic decision-making should incorporate risk diversification. What are the key factors behind such seemingly political risk-seeking behavior?

As a typical country risk, political risk, sometimes refers to geopolitical risk, is the risk that investment returns may suffer from political changes or turbulence in a country. The instability that affects investment returns may result from changes in governments, legislatures, other foreign policymakers, or military control institutions. Evidently, political risk is becoming increasingly important in today's transnational economic and trade activities because of the trade wars and COVID-19 pandemic. The classical country risk theory measures political risk from the perspective of a hypothetical “average person.” In other words, all investors from different countries are assumed to face exactly the same political risk in the host country, which is the main reason why classical theory cannot explain some real phenomena. For example, China's OFDI and project contracting decisions mentioned above, as well as particular Chinese investment projects, are banned in some countries.

Actually, the country relations are extremely important in the decision-making of international economic and trade activities. Although it is not always the decisive factor, it can strengthen or weaken the effect of other influencing factors. Stable and friendly political relations, past cooperation experience, and cultural proximity among countries can enhance investor confidence, reduce investment uncertainty, and have a positive impact on investment choice. In practice, positive country relations can break through geographical constraints, economic gap, and cultural distance, and greatly improve the breadth and depth of economic and trade cooperation between the two countries, while poor country relations make investors have to give up their projects in spite of superior market conditions of the host country.

From the longitudinal perspective, the country relations are of historicality and variability. The historicality refers to the accumulation of bilateral relationships over time, both positive and negative ones. The past and current friendly relationships can drive more exchanges and interactions in the future, so that the relationships will be continuously consolidated and there will be a certain type of inertia, forming a virtuous cycle. The variability refers to the sudden occurrence of conflicts, and the friendship may immediately cool down or even freeze.

From the transverse perspective, country relations are the comprehensive result of economic, political, social, and cultural interactions between countries. Political and economic relations influence each other and generally dominate the country relations, while social relations evolve in a subordinate way. This is the complexity of country relations. “The Belt and Road Initiative” proposed by China, for example, put forward the overall layout of policy coordination, connectivity of infrastructure, unimpeded trade, financial accessibility, and people-to-people bonds, which from the perspective of the country relations are to enhance economic relations as the guidance, to strengthen political relations as assistance, while improving the people's exchange and friendship. Thus, the country relations will be improved further and will have a very positive impact on economic cooperation. It may be because of the historicality, variability, and complexity that the quantitative analysis of country relations is quite difficult and hardly seen in the literature. In contrast, the analysis of unilateral environmental factors of host countries is much easier. In order to study the rationale behind complex decision-making in foreign economic and trade cooperations, it is necessary to investigate the measurement of country relations.

This article explores an evaluation framework of country relations from the aspects of politics, economy, and society, based on the historical interactions, cooperation, and exchanges between two countries. The evaluation results can be applied to the decision-making analysis of international trade, transnational investment, and project contracting.

## 2. Literature Review

When studying the development and change of foreign economy and trades, location choice, and other issues, many scholars have taken into account the influence factors of both the home and host countries. For instance, the trade gravity model takes the economic sizes of the two countries as positive factors and the geographical distance of the two countries as a negative factor. This basic model and its extensions, which constantly incorporate market level, resource endowment, cost, risk, and other factors, can better explain the changes in the development of foreign economic trades [8–15]. Those factors can be classified into political relations, economic relations, social aspects, and others.

Politics-related bilateral factors mainly include the political connections and interactions as well as the differences in institutional management between the two countries. Li [16] utilized the “event data analysis” method and introduced a “conflict-cooperation model” for the study of international relations. Yan and Zhou [17] argued that the relational scores should be equal to the one-period lagged scores plus the impacts of the current period events, and the marginal effect of the new events could vary with the current relation status. Ma et al. [18] adopted the key factors accumulation method, including eight key factors, which improves the comparability between different types of events and consistency of scores. Knill et al. [9] measured the bilateral political relations by UN voting inconsistency. Zhang et al. [19] clarified the theoretical mechanism of the interaction effect between them, including four aspects of bilateral political relations. There are also many studies on OFDI decision-making from the perspective of institutional distance and corruption distance [20–23].

Bilateral factors related to the economy are mainly the economic and trade cooperation in the past and the difference between the economic development levels. Chen and Li [24] studied the influence of geographical distance, institutional distance, economic distance, and cultural distance on location choice in “The Belt and Road” countries' international production capacity cooperation. Shi et al. [25] discussed the influence of distance to the multinational enterprise host selection decisions and established a national distance model. Blanc-Brude et al. [26] verified empirically that economic distance could explain FDI location better than geographical distance and administrative distance. One can also see more discussions on the relationship between economic distance and FDI in Cui and He [27].

Bilateral social factors include population movements between the two countries and the differences in language, religion, culture, *etc*. Based on the Hofstede cultural dimensions, Kogut and Singh [28] defined cultural distance by a normalized Euclidean distance squared. Yin and Lu [29] analyzed the complex nonlinear relationship between cultural distance and international direct investment. Yan and Li [10] found empirically the relation between location choice of Chinese enterprises and country risk, cultural difference, market size, etc. Slangen and van Tulder [30] pointed out that cultural distance and political risk are suboptimal, while the governance quality of foreign countries is a better proxy for external uncertainty. Based on the World Values Survey (WVS), Gustavode et al. [31] determined the cultural distance between countries using cluster analysis with the Euclidean metric. Beugelsdijk et al. [32] tested the impact of home-host national cultural distance on foreign affiliate sales and found the moderating role of cultural variation within host countries. Tang [33] argued that the cultural distance in individualism encourages bilateral FDI activities, while the power distance does not. There are also other studies on the influences of cultural distance on international economic and trade activities [34–38].

Other frequently considered bilateral factors are geographical distance, knowledge distance, and colonial relations. In Bailey and Li [39]; the geographical distance is defined as the greater circle distance of the geographic center of the two countries. Gao [40] and Xu et al. [41] measured the geographical distance by the straight-line distance between national capitals. Aggarwal et al. [42] studied the impact of geographical distance and cultural distance on foreign portfolio investment using the gravity model. Chen et al. [43] studied the national distance and selected the dimensions of geographical, cultural, institutional, and economy for research. Ghemawat [44] put forward the four dimensions of the cultural, administrative, geographical, and economic distance between countries. Liu et al. [45] comprehended several national distance factors from the aspects of geographical, cultural, economic, political, knowledgeable, diplomatic, and global connective. Drogendijk and Martin [46, 47] determined the country distance index from three basic dimensions: physical distance, socio-economic factors, and cultural and historical linkages. In addition, other scholars have studied the influence of corruption distance, institutional distance, psychological distance, migration, and historical relationship on FDI [48–54].

The measurements of different bilateral factors can be quite different. Bilateral political relations are usually calculated by event-history analysis on political behaviors, leaders' visits, mutual comments, joint engagement in international organizations and military actions. Economic distance is usually calculated by the differences in economic indicators between the two countries. Although the geographical distance is defined as the distance between national capitals, the distance between important ports is a good alternative. In most previous studies, cultural distance is calculated based on the Hofstede cultural dimension data or WVS value survey data. The institutional distance is calculated with the Corruption Perceptions Index (CPI) or the Worldwide Governance Indicators (WGIs).

Now, let us comb through, sort out the indicators, and specify some of the terminologies in the literature. The bilateral indicators defined by the difference between the two countries' individual indicators are often called distances. Both country distance and country relations are bilateral indicators, but the difference is that country distance only considers the comparison of the situation of the two countries, while country relations are the exchange between the two countries. If no distinction is made, as in the existing literature, only the country distance is usually considered, and it may be easy to overlook the importance of country relations. Here, we would like to highlight that this may or may not differ from the conventional concept of distance in mathematics. For example, the economic distance refers to the difference between the levels of economic development in the two countries, while the cultural distance is usually calculated by the European distance using the Hofstede cultural data. Indicators are called relations if they are derived from the interactions between home and host countries. For example, the number of high-level exchanges and interaction between the two countries is scored and used to measure bilateral political relations. The historical import and export volume of the two countries is used to measure the bilateral economic relationship.

As Figure 1 shows, let A and B be the home country and the host country, respectively, and *x*_A_ and *x*_B_ represent certain individual indicators of the two countries, respectively. The indicator *f*(*x*_A_, *x*_B_) derived by a certain kind of difference between *x*_A_ and *x*_B_ is called distance. In addition, let *x*_AB_ be a bilateral interaction between the two countries. A bilateral relationship can be measured by a certain function *g*(*x*_AB_) of *x*_AB_.

Having combed the indicators and clarified the concepts of relations and distance, we find that the relation indicators in the literature mainly include bilateral political relations and diplomatic relations, which lay more emphasis on political aspects, and less on economic and social relations. We argue that historical economic exchanges and cooperation are a foundation for future cooperation, and civilian interaction and exchanges play a non-negligible role in country relations, which are usually treated as exogenous environmental variables in overseas investment decision-making. In fact, the dependence of the host economy on the home country and the civilian relationships can greatly increase foreign investors' confidence. In turn, the home country's investment and engineering contracting can further promote the country-to-country relations. Hence, the economic and civilian relationships must be incorporated in the research of country relations.

## 3. Model and Evaluation

### 3.1. Evaluation Framework and a Simplified Model

We propose a theoretical framework for country relations evaluation with three primary indicators of political relations, economic relations, and social relations. The principles of the secondary and tertiary indicator selection are continuous observability, universality, all-sidedness, and relativity as well. Here, continuous observability means that the data are time series. Universality requires that the selected indicators apply to most country-to-country relations. For this reason, the indicators of colonial relations and common currencies are incorporated with dummy variables in our article. All-sidedness means the inclusion of all or nearly all elements or aspects. For example, the indicator of high-level exchanges and interaction should be extended to include common international networks and organizations. Relativity refers to dimensionless relative measurements for economic relations and social relations, such as differences and/or ratios. Suppose that country A is the largest trading partner of country B, while B is not the largest trading partner of A. The economic dependence of B on A is clearly higher than that of A on B. We use trade and FDI shares, instead of volumes and amounts, to measure the economic relations.

The political relations are stipulated by five subindicators. They are high-level exchanges and interaction, relationship statements, international cooperation, political conflicts, and colonial relations. Among them, the relationship statements are the foundation, the frequent high-level exchanges and interaction reflect the activity, international cooperation reflects the extent of the relation, and political conflicts assess the impact of negative events. The indicator of high-level exchanges and interaction includes four levels, that is, mutual visits of heads of state, meeting of heads of state in a third country, mutual visits of prime ministers and ministers of foreign affairs, and meeting of prime ministers and ministers of foreign affairs in a third country. As to political conflicts, being negative events, we also define four levels in the light of Ma et al. [18]: lowering of diplomatic level, serious military conflict, minor military conflict, and declared protest attitude.

Generally, the effect of political events diminishes gradually because memory fades due to the mere passage of time, as per the decay theory in psychology. Such a decay effect has not been incorporated into the event studies on country relations up to now. We take it into consideration in our model with an attenuation coefficient. See Section 3.2.

The indicators of international cooperation allow to consider the bilateral relations in the context of multilateral interaction. The joint participation in important international organizations is conducive to enhancing cooperation between the two countries under consideration, such as in the Shanghai Cooperation Organization, the ASEAN Regional Forum, the G20, and BRICS, which have greatly boosted political and economic exchanges among participating countries.

The indicator of relationship statements on bilateral relationships includes the full diplomatic relations, which manifests stable medium to long-term country relations, and other joint statements on relation augmentation. Four levels of relationship are considered in this article to reflect the different strengths of the relationship between the two countries. The time length of the existence of the relationship is also incorporated into our model to reflect the degree of consolidation of relations.

The indicator of economic relations, there are seven secondary indicators, including the share of imports, the share of exports, the share of FDI, the share of OFDI, the closing of trade ports, the raising of tariffs, and common currencies. The negative subindicators of economic relations are sorted out from the positive ones. The positive economic indicators represent the degree of economic exchanges between the two countries, measured with the shares of bilateral trades and investment in the total of that of each country. The negative subindicators embody events such as closing trade ports and raising tariffs.

The indicators of social relations include the share of entries, share of exits, and ethnic conflicts. For the social relations, the positive indicator is defined by the total flows between citizens of the two countries, while the negative indicator represents the negative social events occurred in the host country against the home country, such as protests and product boycotts.

The structure of our simplified model of country relations is shown in Figure 2.

### 3.2. Indicator Measurements

Throughout the article, the symbols for the first-level indicators are *P* for political relations, *E* for economic relations, and *S* for social relations.

The political relations indicators of high-level exchanges and interaction and political conflicts are measured using the event analysis method. For the details, one can see the conflict-cooperation model proposed for quantitative analysis of Sino-US relations during the eight years of Clinton's administration [16] and the improved scoring method of country relations in the work of Yan and Zhou [17].

Table 1 shows the indicator system, and Table 1data that will be used. The valuation process can be described as follows.

As pointed above, the attenuation of the effects of political events must be incorporated. The simplest way is to make use of the famous Ebbinghaus method, also known as the Ebbinghaus forgetting curve [55]. Suppose an event occurs at time 0. The attenuation coefficient, denoted by *A*_*t*_, is defined as the proportion of the event effect preserved in people's memory, providing no interference. The attenuation coefficient in Wozniak et al. [55] can be rewritten as follows, where the unit of time is *year*:

(1) $$\begin{array}{c} A_{t}\left\{\begin{array}{cc} 1, & t=0\text{;}\\ 1.84{\left[\log\left(t\right)+\log\left(525600\right)\right]}^{1.25}, & t\;=1\text{,}2\text{,}...\text{,}T.+1.84. \end{array}\right) \end{array}$$

Let *A*_0_ be the scores for bilateral interactive events occurring at time 0. The residual effect in year *t* is equal to *A*_*t*_·*A*_0_. The real effect attenuated of positive events may differ from that of negative events. For simplicity, we assume the symmetry between the two kinds of attenuation.

#### 3.2.1. High-Level Exchanges and Interaction

Four levels of high-level visits and interaction are collected here. The first level refers to visits by heads of state to each other's countries; the second level refers to meetings between heads of state in a third country when participating in international affairs; the third level refers to visits by prime ministers or foreign ministers to each other's countries; the fourth level refers to meetings between prime ministers or foreign ministers in a third country when participating in international affairs. According to the level and importance represented by the four cases, the lowest level is assigned 0.2, and the score is doubled when the level raised by one level, so the four levels are assigned 1.6, 0.8, 0.4, and 0.2, respectively. The scores correspond to the importance level of the event, as shown in Table 2.

Let *n*_*lt*_ be the times of high-level exchanges and interaction at level *l* in year *t*, and *hle*_*l*_ be the event scores, *hle*_*l*_ ∈ {1.6, 0.8, 0.4, 0.2}, *l* = 1, 2, 3, 4. The scores of high-level exchange and interaction *P*1 in year *t* can be computed by

(2) $$\begin{array}{c} P1_{t}=\sum_{l=1}^{4}n_{lt}\cdot hle_{l}\text{,}\;\forall t,t=0,1,\ldots ,T. \end{array}$$

The status of the political relations at *T* is equal to the cumulative residual scores of the high-level exchanges and interaction during the observation periods:

(3) $$\begin{array}{c} P1_{T}^{*}=\overset{T}{\underset{t=0}{\sum }}A_{t}\cdot P1_{t},\;t=0,1,2,\ldots ,T, \end{array}$$

where *A*_*t*_ is computed from (1).

#### 3.2.2. Relationship Statements

Different official statements of country-to-country relations represent different degrees and characteristics of cooperation. The indicator value can be determined according to the statement of the relationship. Pan and Jin [56] set the value of the partnership country equal to 3, cooperative relationship to 2, diplomatic relationship to 1, and no diplomatic relationship to 0. Zhang et al. [19] set the comprehensive strategic partnership of cooperation and comprehensive strategic partnership equal to 3, the strategic partnership of cooperation and strategic partnership to 2, the comprehensive cooperation partnership or partnership to 1, and other relations to 0. Men and Liu [57] grade the relationship statements by three levels, all-weather, strategic, and general. Those authors classified the country-to-country relationship expressions into several different levels, and each level reflects a certain degree of relationship.

For the purpose of method demonstration, we analyze all usual relationship expressions of China with countries established diplomatic ties. As of 14 July 2020, 177 out of 192 countries have established diplomatic relations with China. There are 19 kinds of relationship expressions containing 12 keywords of different frequencies.  Table 3 displays all those relationship expressions and keywords.

These keywords stand for the scope, depth, and mode of cooperation between countries and can be classified into several levels. A relationship expression is usually a combination of several keywords. A change of the keyword combination implies an upgrade or an update of the relationship expression. By decomposing keyword, scoring each keyword, and reconstructing the expression, we can score each of the relationship expressions. This makes our scoring method more flexible than the direct assignment of scores to each relationship expression. The latter approach is used in almost all previous articles on the issue. The scores of the keywords are shown in Table 4. For any relationship expression, the score of each keyword involved can be found in Table 4 and then summed up to obtain the score of the relationship expression.

Generally, a bilateral relation statement can be regarded as a political event. Its influences will gradually diminish if there is no recall. Let *re*_*l*_ be the scores of the keywords of a relationship expression at level *l*, *re*_*l*_ ∈ {0, 1, 2}. The scores of that expression declared *P*2 in year *t* is

(4) $$\begin{array}{c} P2_{t}=\overset{4}{\underset{l=1}{\sum }}re_{lt},\;\forall t,\;t=0,1,2,\ldots ,T. \end{array}$$

The cumulative score of all relationship expressions declared until the end of year *T* is

(5) $$\begin{array}{c} P2_{T}^{*}=\overset{T}{\underset{t=1}{\sum }}A_{t}\cdot P2_{t},\;\;t=0,1,2,\ldots ,T, \end{array}$$

where *A*_*t*_ comes from (1).

#### 3.2.3. Multilateral Interaction

By virtue of the importance the countries attach to a meeting of international or regional organizations, state leaders of different levels attend the meeting. The multiple interactions can then be scored according to the level of state leaders interacting in the context of meetings of international and regional organizations. We consider the scoring criteria in Yan and Zhou [17] as a benchmark and derive the multilateral interaction scores from it. Multilateral interactions in the context of international or regional meetings differ from bilateral ones since they are less influential with a large number of participants and particularly the important bilateral state leaders' meetings are held in one of the two countries, not in the context of multinational leaders' meetings. In general, the larger the number of members of an international organization is, the weaker the influence of such a meeting on the bilateral relations between members is.

Suppose there are *N*_*t*_ international organizations taken into account in year *t*. Let *m*_*nt*_ be the number of members of organization *n*_*t*_, 1 ≤ *n*_*t*_ ≤ *N*_*t*_, and *io*_*nt*_ be the scores of the state leader's meetings of organization *n*_*t*_. The total scores of the multilateral interactions in a given year *t* are equal to

(6) $$\begin{array}{c} P3_{t}=\sum_{n_{t}=1}^{N_{t}}\frac{io_{nt}}{m_{nt}},\;\forall t,t=0,1,2,\ldots ,T. \end{array}$$

The cumulative scores of multilateral interactions in year *T* are therefore

(7) $$\begin{array}{c} P3_{T}^{*}=\sum_{t=1}^{T}A_{t}\cdot P3_{t},\;t=0,1,2,\ldots ,T, \end{array}$$

where *A*_*t*_ is defined in (1).

#### 3.2.4. Economic Relations

As pointed in Section 3.1, bilateral economic interactions can be measured with shares of imports, exports, FDI, and OFDI between two economies. *E*1_*t*_ denotes the share of imports of the home country from the host country in year *t*; *E*2_*t*_ the share of exports of the home country from the host country in year *t*; *E*3_*t*_ the share of the inward FDI of the host country from the home country in year *t*; and *E*4_*t*_ the share of the inward FDI of the home country from the host country in year *t*.

#### 3.2.5. Social Exchange Indicators

The subindicators of the social relations include the share of entries S1 and the share of exits S2, representing how frequent the host country citizens travel to the home country and how frequent the home country citizens travel to the host country, respectively. For a given year *t*, let entry_*t*_ be the number of trips of the host country's citizens to the home country in year *t*; exit_*t*_ be the number of trips of the home country's citizens to the host country; Outbound_*t*_^host^ be the total number of outbound trips of the host country's citizens, and Outbound_*t*_^home^ be the total number of outbound trips of the home country's citizens. Thus,

(8) $$\begin{array}{c} S1_{t}=\frac{{\text{entry}}_{t}}{{\text{Outbound}}_{t}^{\text{host}}}\text{,}\;t=0,1,\ldots ,T,\\ S2_{t}=\frac{{\text{exit}}_{t}}{{\text{Outbound}}_{t}^{\text{home}}}\text{,}\;t=0,1,\ldots ,T. \end{array}$$

### 3.3. Aggregation of Country Relations Index

It is necessary to point out that the dimensional consistency of all the indicators has been considered in our scoring system; that is, the higher the score of an indicator is, the closer the unidimensional relation is between the two countries.

The sum of all the normalized indicators is a trivial aggregation method, which is based on ordinal information. Its underlying hypothesis of the equi-importance of the indicators is undesirable in general. Another simple and most used method is the weighted additive aggregation. However, the justifiability of the weights is generally burdensome to verify. In addition, the additive aggregation methods are compensatory, that is, poor performance in political indicators can be compensated by sufficiently high values of economic and social indicators. The geometric aggregation is also a simple and less compensatory approach. Of course, one can always adopt noncompensatory aggregations, such as the multicriteria analysis. We do not use the last approach in this article because of only a small dataset available for methodological illustration.

Based on the scored second-level indicators, we compute the scores of first-level indicators with the arithmetic mean and then the aggregate of the overall country relations using both weighted additive and geometric approaches.

In the literature of country risk assessment, political and economic risks are often considered equally important. For example in the country risk reports issued by International Country Risk Guide (ICRG) and Euromoney Country Risk (ECR), political risk and economic-financial risk are of equal weights, while other risks are subordinated to them. The indicator system of Country-Risk Rating of Overseas Investment from China (CROIC) includes five subindicators: economic foundation, solvency, social resilience, political risk, and relations with China, in which the economic indicators (the first two) and political indicators (the third and fourth) are both weighted at 40% while the social resilience indicator is weighted by 20%. In the light of those weighting methods, we set the weights of political relations and economic relations both at 40% and that of the social relations at 20%. The concise calculation method of each index is shown in Table 5, where *R*^+^ and *R*^∗^represent the additive and geometric aggregates, respectively.

**Remark 1 .**

In *R*^∗^, the political relation index is in form of [(1 + *P*)/2], instead of *P*. This allows *P* to take negative values in [−1, 1].

### 3.4. The Initial Value of the Political Relations

Unlike the indicators of economic and social relations, *E* and *S*, which are defined by current year data only, the value of the political relations *P* includes, by the definition, the effect of lagged values cumulative from time −∞. Hence, the true initial value *P*_0_ of *P* is intrinsically unobservable. One can set *P*_0_ equal to zero if the number of observation periods is large enough. In fact, *P*_0_ = ±1 in the extreme cases and the remaining influence of *P*_0_ on *P*_*t*_ is equal to ± *A*_*t*_, which tends to 0. The influence of extreme initial values on *R*_*t*_^+^ is equal to 0.4*A*_*t*_. This implies that any initial value *P*_0_ will create an error in *R*_5_^+^ less than 0.4*A*_5_ ≈ 0.061 and in *R*_10_^+^ less than 0.4*A*_10_ ≈ 0.058. In our case study in the next section, we assume that *P*_0_ = 0. In contrast, *R*^∗^ is more sensitive to the initial value assumption. For this reason, *R*^∗^ is not recommended when the number of observation periods is small.

## 4. Case Study

Let us take China as the home country and measure the relations between China and other BRICS countries. Russia, India, South Africa, and Brazil are important target countries for Chinese outward FDI. The data sources include the Ministry of Foreign Affairs of the People's Republic of China (for the data of high-level exchanges and interaction, relationship statements, and international cooperation), the BRICS Joint Statistical Publication 2018 (for the data of imports, exports, FDI, OFDI, entries, and exits of China to the four countries), the China Statistical Yearbook 2018 (for the data of total imports, exports, FDI, OFDI, entries, and outbound trips of China), the World Bank Open Data, and the Yearbook of Tourism Statistics Data 2012-2016, 2014-2018 (for the data of total outbound trips of the four countries). There is no negative event recorded in our datasets, wherefore the five negative event indicators are set to 0. The calculated results are shown in Table 6.

The chronological evolution of the political relations, economic relations, social relations, and overall country relations *R*^*+*^ and *R*^*∗*^ is shown in Figures 3–7, respectively.

The overall relations of China with Russia are closer than those of China with other BRICS countries. This is consistent with most people's perception. Evidently, the stable China-Russia political relations dominate other relations. Both the additive and geometric aggregates show that the overall relations between China and other BRICS countries can be ranked as China-Russia, China-India, China-Brazil, and China-South Africa. Between China and Brazil, the poorer performance in political and social relations is compensated to a certain extent by the higher values of the economic relations. It is also notable that China-India overall relations are stable although their social relations tend to be alienated.

## 5. Conclusions

Since the relationship between nations could determine the location advantages in the international investment mode selection to a certain extent, this article has studied the evaluation problem of the country relations. First of all, through literature analysis, it was found that the indicators of country relations and distance were often mixed in empirical studies. Therefore, this article distinguished the meanings of each, according to the differences in their reference data, which is the first contribution. Then, based on the fact that the current country relations mainly focused on political relations, this article added economic relations and social relations, and constructed a relatively reasonable analytical framework from three aspects. A simplified framework for the evaluation of country relations was established, and the indicators at all levels were determined according to the theoretical analysis and the requirements of continuous observability, universality, all-sidedness, and relativity of data. At the same time, the quantitative methods of each indicator in the index system were designed and improved. That is the second contribution of the article. Finally, the practicability and rationality of the evaluation model of country relations were illustrated through a case of China and other BRICS countries. The calculated results were easy to analyze and explain, and could reflect the changes of bilateral relations in time, as well as the characteristics and differences of relations in different aspects and different countries.

There are two points in this article that need further discussion and improvement. The first is the further optimization of the index system, because the current index system is based on theoretical and literature analysis and can be supplemented and verified in terms of completeness by organizing expert discussions. Second, more work is needed to compare and verify whether there is a more reasonable weight design of indicators, so as to get the optimal conclusion.

Two related problems are deserved further study. The first is whether there is an interaction between the three aspects of relations and how they work together in international trade and investment. In addition, applying the method proposed in this paper to the study of unreasonable phenomena such as the risk tendency in international trade and investment, such as the investment decision analysis of China in regions of Africa and One Belt and Road countries, we can try to explain some research paradoxes, which will be a meaningful research direction.

## Figures and Tables

**Figure 1:** Data sources and classification of different indicators.

**Figure 2:** Structure of a simplified model for country relations assessment.

**Figure 3:** Political relations between China and other BRICS countries.

**Figure 4:** Economic relations between China and other BRICS countries.

**Figure 5:** Social relations between China and other BRICS countries.

**Figure 6:** Overall country relations (*R*^+^) between China and other BRICS countries.

**Figure 7:** Overall country relations (*R*^∗^) between China and other BRICS countries.

**Table 1:** Indicator system.

First-level indicators	Second-level indicators	Data examined
Political relations	High-level exchanges and interaction	The frequency, leaders, and venue of high-level exchanges and interaction
	Relationship statements	Expression and time of relationship statements
	International cooperation	The number of members of the organizations and the level of attending leaders
	Political conflicts	The frequency and level of political conflicts
	Colonial relations	Whether or not they have colonial relations
Economic relations	Share of imports	Imports from the host country and total imports
	Share of exports	Exports to the host country and total exports
	Share of FDI	FDI of host country and total FDI
	Share of OFDI	OFDI to the host country and total OFDI
	Closing of trade ports	Time and frequency
	Raising of tariffs	Proportion and frequency
	Common currencies	Whether or not they have colonial relations
Social relations	Share of entries	Entries from host country and total outbound
	Share of exits	Exits to host country and total outbound
	Ethnic conflicts	Time, frequency, and degree

**Table 2:** Levels and scores of high-level exchanges and interaction.

Levels	Scores
(1) Heads visit	1.6
(2) Heads meeting in the third country	0.8
(3) Prime/foreign ministers visit	0.4
(4) Prime/foreign ministers meeting in the third country	0.2

**Table 3:** Statistics on the relationship expressions between China and other countries.

Relationship expressions	Number	Keywords	Frequency
Comprehensive strategic partnership	36	Partnership	79
Strategic partnership	12	Strategic	69
Comprehensive strategic and cooperative partnership	10	Comprehensive	58
Comprehensive and cooperative partnership	6	Cooperative	27
Strategic cooperative partnership	4	Friendly	4
Comprehensive friendly and cooperative partnership	2	Reciprocal	2
Friendly partnership	2	Innovation	1
Strategic cooperative partnership	1	Development	1
Innovation comprehensive partnership	1	Coordination	1
Development partnership	1	Global	1
Reciprocal strategic partnership	1	All-weather	1
Comprehensive strategic cooperation relationship	1	All-round	1
Comprehensive strategic partnership of coordination	1		
Global comprehensive strategic partnership	1		
All-weather strategic cooperative partnership	1		
All-round cooperative partnership	1		
Strategic cooperation relations	1		
Strategic reciprocal relations	1		
Total	83		

Source: Ministry of Foreign Affairs of the People's Republic of China. (Quoted on 14 July 2020).

**Table 4:** Keywords and scores of the relationship expressions.

Level	Keywords	Scores
(1) Foundation level	Partnership	2
(2) Cooperative relation	Cooperative, coordination	2
	Friendly, reciprocal	1
(3) Cooperation characteristics	Strategic	2
	Innovation, development	1
(4) Cooperation scope	All-weather	2
	Comprehensive, global	1

**Table 5:** Aggregation of country relation index.

First-level indicators	Second-level indicators	Quantification	Aggregation
*P*	*P*1	*P*1^∗^ = Σ*A*_*t*_·(Σevent score × times of exchanges)	*P* = (*P*1^∗^ + *P*2^∗^ + *P*3^∗^)/3
	*P*2	*P*2^∗^ = Σ*A*_*t*_·(Σkeyword score × number of keywords)	
	*P*3	*P*3^∗^ = Σ*A*_*t*_·(Σmultilateral event score/number of members)	
*E*	*E*1	*E*1 = import/total import of the home country	*E* = (*E*1 + *E*2 + *E*3 + *E*4)/4
	*E*2	*E*2 = export/total export of the home country	
	*E*3	*E*3 = FDI/total FDI of the home country	
	*E*4	*E*4 = OFDI/total OFDI of the home country	
*S*	*S*1	*S*1 = entry/total outbound of the host country	*S* = (*S*1 + *S*2)/2
	*S*2	*S*2 = exit/total outbound of the home country	
*R*	*P*, *E*, *S* = dimension standardization		*R* ^*+*^ = 0.4*P* + 0.4*E* + 0.2*S*
			*R* ^*∗*^ = [(1 + *P*)/2]^0.4^ × *E*^0.4^ × *S*^0.2^

**Table 6:** Overall relations between China and other BRICS countries.

Indicator	Country	2012	2013	2014	2015	2016	2017	2018	2019
*P*	China-Russia		0.36	0.36	0.35	0.36	0.37	0.36	0.35
	China-India		0.24	0.23	0.23	0.25	0.24	0.25	0.26
	China-South Africa		0.20	0.21	0.23	0.20	0.20	0.21	0.19
	China-Brazil		0.19	0.20	0.19	0.19	0.19	0.18	0.20
*E*	China-Russia	0.34	0.32	0.31	0.35	0.31	0.31		
	China-India	0.23	0.20	0.21	0.25	0.25	0.26		
	China-South Africa	0.14	0.19	0.18	0.17	0.17	0.14		
	China-Brazil	0.29	0.29	0.29	0.24	0.28	0.29		
*S*	China-Russia	0.44	0.39	0.43	0.46	0.53			
	China-India	0.35	0.39	0.37	0.36	0.31			
	China-South Africa	0.11	0.12	0.10	0.09	0.08			
	China-Brazil	0.10	0.10	0.10	0.09	0.09			
*R* ^+^	China-Russia		0.35	0.35	0.37	0.37			
	China-India		0.25	0.25	0.26	0.26			
	China-South Africa		0.18	0.18	0.18	0.16			
	China-Brazil		0.21	0.22	0.19	0.20			
*R* ^∗^	China-Russia		2.32	2.33	2.37	2.36			
	China-India		2.18	2.18	2.21	2.19			
	China-South Africa		1.99	1.95	1.93	1.91			
	China-Brazil		2.06	2.05	2.00	2.03			

## Data Availability

The data that support the findings of this study are available from the corresponding author upon reasonable request.
